The article "Impact of the Aversive Effects of Drugs on Their Use and Abuse" was published in 2022. Journal: Behav Neurol.

# Impact of the Aversive Effects of Drugs on Their Use and Abuse

**DOI:** 10.1155/2022/8634176

**Published:** 2022-04-20

**Authors:** Anthony L. Riley, Hayley N. Manke, Shihui Huang

**Affiliations:** Psychopharmacology Laboratory, Department of Neuroscience, Center for Neuroscience and Behavior, American University, 4400 Massachusetts Ave NW, Washington, D.C. 20016, USA

## Abstract

Drug use and abuse are complex issues in that the basis of each may involve different determinants and consequences, and the transition from one to the other may be equally multifaceted. A recent model of the addiction cycle (as proposed by Koob and his colleagues) illustrates how drug-taking patterns transition from impulsive (acute use) to compulsive (chronic use) as a function of various neuroadaptations leading to the downregulation of DA systems, upregulation of stress systems, and the dysregulation of the prefrontal/orbitofrontal cortex. Although the nature of reinforcement in the initiation and mediation of these effects may differ (positive vs. negative), the role of reinforcement in drug intake (acute and chronic) is well characterized. However, drugs of abuse have other stimulus properties that may be important in their use and abuse. One such property is their aversive effects that limit drug intake instead of initiating and maintaining it. Evidence of such effects comes from both clinical and preclinical populations. In support of this position, the present review describes the aversive effects of drugs (assessed primarily in conditioned taste aversion learning), the fact that they occur concurrently with reward as assessed in combined taste aversion/place preference designs, the role of aversive effects in drug-taking (in balance with their rewarding effects), the dissociation of these affective properties in that they can be affected in different ways by the same manipulations, and the impact of various parametric, experiential, and subject factors on the aversive effects of drugs and the consequent impact of these factors on their use and abuse potential.

## 1. Drug Use and Abuse

According to recent results from Monitoring the Future (MTF, 2021), a national survey on drug use by 8^th^, 10^th^, and 12^th^ graders, 27.3% of students (averaged across grades) reported use of illicit drugs in the past year [1] (for more recent unpublished findings, see https://www.drugabuse.gov/drug-topics/trends-statistics/monitoring-future). In a sample of participants aged 12 years and older in 2020, the National Survey of Drug Use and Health (NSDUH, 2020) found that 13.5% used an illicit drug in the past month [2]. These surveys clearly indicate that a variety of drugs are used, but importantly, they also indicate that a smaller subset of individuals abuse these same drugs. For example, MTF reported patterns and amounts of drug intake generally associated with abuse. Specifically, daily marijuana prevalence in 2020 was at 1.1%, 4.4%, and 6.9%, and binge drinking (defined as at least 5 or more drinks in a row at least once in the past two weeks) was at 5%, 10%, and 17% for 8^th^, 10^th^, and 12^th^ graders, respectively [1]. Related findings have been reported by the NSDUH that found that 40.3 million people had a past year substance use disorder [2] as defined by the *Diagnostic and Statistical Manual of Mental Disorders (DSM-5)* (see [2] for the basis of the dramatic difference in the rates of drug abuse when diagnoses are based on the DSM-4 vs. the DSM-5). Further, according to the World Drug Report (2021), the Global Burden of Disease Study (GBD) in 2019 found that substance use disorders accounted for the largest portion of disability-adjusted life years (DALYs), a measure of disease burden taken from the combination of both the number of years of life lost because of premature death and the number of years of life lived with disability [3]. In fact, drug use disorders accounted for 59% of DALYs with approximately 18.1 million years of “healthy” life lost due to disabilities or premature death [3]. Interestingly, among people aged 12 or older, only 1.4% received any treatment for substance use [2].

## 2. Allostatic Model of Drug Use and Abuse

Given the multiple causes and consequences of drug use and abuse, understanding this complexity is critical to prevention and treatment strategies [4]. One comprehensive model of these issues has recently been presented by Koob and his colleagues who describe the various stages of drug use and abuse, the factors important in their display, and the neurobiological substrates of each (as well as the role of these substrates in the transition from use to abuse, drug maintenance, and relapse; see [4–7]). Specifically, Koob and his colleagues describe a neuroadaptation model of addiction that consists of three distinct stages: binge/intoxication, withdrawal/negative affect, and preoccupation/anticipation, which differ significantly between acute and chronic drug use (see Figure 1).

Acute use represents a pattern of drug intake in the majority of the population using drugs (roughly between 85 and 90%) that is more impulsive and controlled. Application of Koob's model to individuals in this group reveals a specific characterization of the effects of the drug (binge/intoxication), the affective state of the individual following the cessation of the drug effect (withdrawal/negative affect), and the subsequent desire for the drug in its absence (preoccupation/anticipation). As noted in Figure 1, for acute use (the impulsive condition), the drug itself is rewarding, generating an effect preferred by the user (i.e., a rewarding effect). After the drug's effects have subsided, there is no change in the user's affective state, i.e., the user is relatively neutral in the drug's absence. Finally, there is no true craving for the drug in this group, but if such anticipation of the drug does occur, it is one of a desire to repeat its rewarding effects. Importantly, the drug does initiate a compensatory response (allostasis) that generally is opposite in nature to that of its initial effect. If the user takes the drug relatively infrequently, at low doses, and by routes of administration that have a slow onset and offset, this allostatic state subsides and there is no appreciable change in the abovementioned characterization. The drug maintains its reinforcing effects with little change with its absence and no appreciable craving.

However, if the pattern of drug use changes, e.g., increased frequency of use at higher doses and by routes of administration with more rapid onset (and offset), neuroadaptations occur that drive the transition from use to abuse (involving roughly 10-15% of individual drug users). These neuroadaptations move impulsive use to compulsive use where an individual loses control over abstaining from the drug, escalates drug intake, and relapses [5]. For this group of individuals, the drug may still have positively reinforcing effects, although they are likely to be diminished as a result of the drug-induced downregulation of mesolimbic and mesocortical pathways [7] that mediate these effects. This tolerance induces escalation of drug intake. Further, because these systems are involved in regulating natural reward, their diminished state (a compensatory reaction to elevated drug intake) results in a negative affect (anhedonia-dysphoria, anxiety, irritability, and sleep disturbances) when the drug is no longer present. This negative affect drives further drug intake by negative reinforcement which is exacerbated by sensitized brain stress systems (primarily in the extended amygdala, i.e., central nucleus of the amygdala, the bed nucleus of the stria terminalis, and a transition zone in the nucleus accumbens) that reflect further compensation to elevated intake. Finally, these individuals now crave the drug when it is absent as the negative affect grows with time since taking the drug. Intake is increased as well by neuroadaptations in yet other systems, e.g., orbitofrontal cortex, which normally mediates salience for traditional reinforcers such as food and sex, is now shifted toward the drug, and the systems involved in executive function (prefrontal cortex; planning, inhibition, memory, and attention) are downregulated. Consequently, these individuals have difficulty targeting relevant reinforcers and inhibiting further drug intake. The cycle continues and spirals out of control with escalated intake, more frequent use, and high rates of relapse (potentiated by the presence of cues and stress that reactivate the mesolimbic and cortical areas via increased input from the frontal cortex).

## 3. Role of Reward in Drug Use and Abuse

The addiction cycle proposed by Koob and his colleagues [5, 7] illustrates how drug-taking patterns transition from impulsive (acute use) to compulsive (chronic use) as a function of neuroadaptations leading to the downregulation of dopamine pathways and processes, upregulation of stress systems, and the dysregulation of the prefrontal cortex (see above). Important to this analysis is that although the nature of reinforcement initiating and mediating these effects differs (positive vs. negative), the general role of reinforcement in drug intake (both acute and chronic) is well characterized [9–12]. However, drugs have other stimulus properties that may be important as well in drug use and abuse. One such property is a drug's aversive effect that limits drug-taking instead of initiating and maintaining it. The evidence for such effects comes from both clinical and preclinical research (for an excellent review of how initial responses to a drug impact subsequent use in both clinical and preclinical populations, see [13]).

## 4. Clinical Evidence of the Aversive Effects of Drugs of Abuse

Clinical anecdotal reports note that drugs have both rewarding and aversive effects (with their use a function of the balance of these two properties; see [14] for a discussion; for factors impacting drug intake, see [9, 13, 15]). For example, smokers often report the first exposure to nicotine as aversive (heart palpitations, feeling faint, dizziness, throat irritation, coughing, and nausea) and adjust their intake to reduce these effects or as tolerance develops allowing them to continue to smoke. Interestingly, DiFranza and colleagues [16] noted that among first-time users (primarily young adolescents), throat irritation with the first puff is a predictor of reduced cigarette use whereas relaxation, dizziness, and nausea predict subsequent cigarette use disorder (see also [17, 18]). In a self-report of the effects of mescaline, the user described vivid hallucinations but noted aversive side effects such as nausea and dizziness that led to speculation that the drug would not likely become popular given that such side effects would spoil the generally positive effects of the drug [14]. One also sees these aversive effects with injected heroin as the drug has been reported to induce an orgasmic rush that is often accompanied by nausea, retching, and vomiting. These aversive side effects diminish with repeated dosing [19]. Effects of caffeine have also been reported to reflect the interaction of its rewarding and aversive effects, and this interaction appears to be dose-dependent. For example, in an assessment of intake and reactions to varying doses of caffeine, low doses (e.g., 100 mg) were found to be positively rewarding to all subjects (with none reporting any negative effects). With increases in dose, a general preference for the drug decreased as specific aversive or unwanted effects such as jitteriness and nervousness appeared [14]. Similar dose-related effects have been reported with phencyclidine (PCP). For example, at low doses, PCP produces a rewarding effect that is often accompanied by a range of aversive effects, e.g., thought disturbances, as well as violent behavior. With even greater doses, the aversive and unpleasant side effects such as panic, fear paranoia, incoherent speech, and bizarre behaviors become more intense that may dimmish the likelihood of further intake (see also [15, 20]).

Work with alcohol further demonstrates the aversive effects of drugs and how these effects modulate or impact drug intake. For example, the mutation in the gene coding for the enzyme aldehyde dehydrogenase (from the typical isozyme ACDH2 to the less efficient isozyme ACDH2∗2; found predominately in East Asian populations) results in the reduced ability to metabolize acetaldehyde, a metabolite of alcohol [21]. Acetaldehyde has been reported to produce a variety of adverse reactions, e.g., flushing of the face, headaches, and heart palpitations (with the severity of these reactions greater in individuals homozygous for the ACDH2∗2 gene), and appears to be protective against further alcohol intake among those with the gene for this enzyme (see [22]; for evidence of acetaldehyde's rewarding and motivating effects, see [23]. The use of the drug disulfiram, a drug that blocks the metabolism of acetaldehyde, in the treatment of alcoholism is based on this same principle.

In an assessment of patterns of alcohol intake in humans, Baker and Cannon [24] noted that approximately 45% of individuals hospitalized for the treatment of alcoholism reported aversions to the flavor of specific alcohol preparations most of which were acquired as a function of overconsumption during early adolescence. That is, becoming sick with their initial alcohol experience limited subsequent consumption of those specific beverages. Similarly, based on a survey of taste aversions in humans, Logue et al. [25] reported upwards of 25% of 517 individuals who answered the survey indicated aversions to alcohol that were associated with earlier patterns of alcohol consumption. It is interesting in this context that one chemical treatment of alcoholism utilizes aversion therapy in which alcohol consumption is associated with an injection of a nauseant drug that induced aversions to the taste of alcohol ([26–28]; for reviews, [29, 30]). Further (and along the lines noted above with genetic mutations), individuals appear to be differentially sensitive to these aversive effects of alcohol evidencing another genetic vulnerability, in this case toward greater consumption in those individuals less affected by alcohol's aversive effects. Importantly, these vulnerabilities appear to interact with experience as well given that individuals who do not initially experience aversive effects seem to be protected from subsequent aversive reactions (either through tolerance to alcohol or the added rewarding effects of alcohol in ameliorating withdrawal symptoms; see [24]).

These data from clinical populations illustrate that drugs of abuse are complex pharmacological agents that possess multiple stimulus effects, with the rewarding effects increasing vulnerability to initial use and subsequent abuse and the aversive effects limiting intake. Such effects can occur at the same dose; some are dose-dependent. Some effects appear to be impacted by genetic vulnerabilities; some are affected by experience. Independent of the drug and the factors that modulate its effects, what is clear is that individuals weigh the balance of these effects and intake is either adjusted or continued with the anticipation that the aversive effects will be lessened with use (tolerance) or will become less salient as the rewarding effects increase (sensitization).

## 5. Preclinical Evidence of the Aversive Effects of Drugs of Abuse: Taste Aversions

Work with preclinical populations also reports evidence of aversive effects of drugs of abuse. While there is considerable support for such effects in preclinical literature, the roots of this evidence are in toxicology [31]. In fact, work demonstrating such effects came from investigations related to military applications during World War II, i.e., the effects of toxins on rodent infestations (see [32]) and the effects of radiation exposure on biological systems (see [33]; for a review, see [34]). Initial field trials on rodent management with baits (i.e., a poison mixed with food base) presented a major difficulty, as rats exhibit a neophobic response toward novel foods and rarely sample enough of the bait to ingest a lethal amount of the poison. In early studies of this phenomenon (bait-shyness), Rzóska [32] fed rats a food base laced with poison and noted that rats that had initially accepted the poisoned bait avoided the same bait in successive trials, but when a new base laced with the same poison was offered, they readily consumed the new bait. In speculating on these empirical findings, i.e., refusal of identical poisoned bait and acceptance of experienced poison in the new base, Rzóska concluded that the rats associated the food base, rather than the poison itself, with the illness experienced following ingestion of the bait so they avoided the same food on subsequent trials.

In the early 1950s, this phenomenon of associative learning between a novel taste and illness was further demonstrated with the effects of radiation by Garcia and his colleagues who observed that rats given water in plastic bottles during radiation exposure subsequently avoided drinking water from those plastic bottles. Importantly, the same rats would drink the water provided in glass bottles, suggesting that the plastic bottle gave the water a unique taste that was associated with the effects of radiation (for a history of Garcia's early work with radiation, see [34]). In subsequent studies, Garcia and colleagues [33] tested the basis of these aversions by giving rats a novel saccharin solution to drink during radiation exposure and reported that those rats strongly suppressed consumption of the saccharin solution after a single pairing of saccharin with radiation compared to the control group that was not exposed to radiation following intake of the saccharin. Garcia et al. concluded that the aversive effects of radiation conditioned an aversion to the radiation-paired flavor (see Figure 2). This initial report demonstrated the fast and robust nature of conditioned taste aversions (CTAs) as a form of classical conditioning, wherein learning occurred with a single pairing; the aversion was dose-dependent (30 vs. 57 roentgen (r)) and evident for over 30 days post conditioning despite the fact that animals were given continuous access to the initially preferred saccharin solution and water during this period. Such aversions have been reported to be maintained with a year (53 weeks) intervening between its acquisition and eventual test [35].

Subsequently, Garcia et al. [36] demonstrated that an aversion to saccharin was acquired with an interstimulus interval as long as 75 min (i.e., when the delay between consumption and radiation was 75 min). In a separate study published the same year, taste aversion learning appeared selective to gustatory stimuli, wherein rats selectively associated saccharin with radiation but audiovisual cues with foot shock [37]. These unique conditions under which CTA was acquired, that is, learning with one trial, over long delays and relatively selective to tastes, led to the reconceptualization of the role of evolution in shaping behavior and learning. It seems plausible that natural selection favored organisms able to quickly learn the taste-illness association. Given that aversive outcomes are likely to occur after some delay as the natural function of digestion, the ability to learn a taste-illness association over long delays prevents repeated consumption of toxic foods. Such adaptive specialization for survival also extended to the selective nature of CTA learning that prevents irrelevant stimuli (e.g., external cues) from interfering with the learning of a taste-illness association [38–40].

## 6. Taste Aversions as an Index of Toxicity

Although the initial investigations into CTAs primarily focused on their empirical assessments and theoretical implications, subsequent research in this area shifted to explore the conditions under which CTA learning can be acquired, effects of various manipulations on its expression, and issues of mechanisms and applications. An important extension involved the use of CTA preparation as a tool to detect and characterize the behavioral and physiological effects of a toxin [31]. Empirically, the application of CTA as an index of toxicity is supported by the evidence that a wide range of classical toxins that were characterized by other behavioral and pharmacological tests could also condition taste aversions under various experimental conditions (for a review, see [31]). For example, Nachman and Hartley [41] demonstrated that various rodenticides highly toxic to rats (i.e., copper sulfate, red squill, and sodium fluoroacetate) produced strong taste aversions often with only a single pairing of a novel taste with the compound. In addition to being rapidly learned, CTAs appeared relatively sensitive to detecting the aversive effects of drugs relative to other indices of toxicity. For example, trimethyltin, a known neurotoxicant that causes specific damage to the hippocampus, induces taste aversions [42, 43]. In more traditional behavioral assays, a single administration of trimethyltin disrupts hippocampus-dependent performance as measured in a number of tasks, e.g., Hebb-Williams maze, radial-arm maze, and differential reinforcement of low rates of responding (DRL). Interestingly, the dose of trimethyltin needed to condition a taste aversion is 500% less than that required to produce effects in other behavioral indices of toxicity [42, 43]. These dose-response comparisons substantiate the taste aversion design as a sensitive index in detecting toxicity, as compounds that support taste aversions generally do so at lower doses than are necessary to produce effects in more traditional assessments of toxicity. From a theoretical perspective, the sensitivity of the taste aversion design appears to be a natural extension of the concept of adaptive specialization in normal consummatory behavior. An organism that can learn the toxic potential of its food source is likely to quickly avoid subsequent toxicosis and reduce the possibility of ingesting the fatal dose of the toxin (see above). Research investigating other compounds with toxic and adverse effects within the CTA preparation steadily increased throughout the 1970s with several well-known toxins such as barium sulfate, cyanide, red squill, strychnine sulfate, and sodium fluoride reportedly producing CTAs (for a more comprehensive list of compounds with toxic and adverse effects that induce CTAs, see Table 1). Although most classical toxins (and neurotoxins) reliably condition taste aversion, several compounds with known toxicity have been reported to be ineffective. While such caveats clearly suggest a limitation of the CTA preparation as an index of toxicity, alternative interpretations have been raised in relation to specific procedures in assaying taste aversions that might account for these failures (see [31] for a discussion of the basis for the failure of known toxins to condition taste aversions and procedural variations of the CTA preparation that could increase the efficacy of those compounds to induce CTA).

There are certainly other behavioral assays for the aversive effects of drugs than taste aversion learning, e.g., suppression of normal regulatory behavior (food and water intake) and disruptions of scheduled-controlled responding, activity, learning and memory, and hedonic shifts (see Riley and Tuck, 1985 [31]). One assay very related procedurally to conditioned taste aversions is the conditioned place aversion (CPA) preparation in which specific environments (or contextual cues) are associated with drug injection. In this preparation, animals avoid or spend less time in the drug-paired environment than in one that is paired with the drug vehicle. Although this procedure is often used to assess the aversive effects of a drug, it should be noted that when direct comparisons have been made between the taste and place aversion designs, aversions are generally more rapidly acquired and more strongly evident in taste (than place) conditioning (for a direct comparison between LiCl-induced taste and place aversions and a review of other drug comparisons in these two designs, see [99]). These differences between the taste and place conditioning procedures in such assessments are likely a function of the relatively greater associability of taste (over place) in the conditioning of aversive effects (see [38–40]). It is important to note that the majority of drugs of abuse that reliably induce taste aversions fail to induce a place aversion (in fact, generally inducing a place preference; see below) or produce a CPA under specific parametric conditions (high doses, without a drug history, and time of injection relative to placement in chamber) or with specific sex, age group, or species (for a discussion, see [99]). Given that taste aversion conditioning has been more extensively examined as a behavioral assay of the aversive effects of drugs and does so with greater sensitivity and generality, the present review focuses primarily on conditioned taste aversion learning in our analysis.

## 7. Conditioned Taste Aversions Induced by Drugs of Abuse

Although the initial work on the conditions supporting taste aversion learning assessed compounds with adverse or toxic effects as potential aversive stimuli, by the early 1970s, a host of other compounds were being investigated, some of which included drugs of abuse. For example, Lester et al. [100] assessed taste aversion learning with ethanol in which male Wistar rats were given 10 min access to a saccharin solution that was then followed by administration of ethanol (at various concentrations and doses and by different routes of administration). Under these parametric conditions and with only a single conditioning trial, ethanol induced significant suppression of saccharin consumption, and as reported with work with known toxins [34], the degree of the aversions induced was dose-, concentration-, and route-dependent. Importantly, control subjects receiving the same saccharin solution paired with injections of the ethanol vehicle readily consumed it, indicating that the suppression evident in the ethanol-treated animals was a function of the association of saccharin with ethanol.

The following year, Cappell and LeBlanc [101] assessed the aversive effects of several other drugs of abuse, specifically mescaline and d-amphetamine. In the assessment with mescaline, male Wistar rats were given access to a novel saccharin solution and injected intraperitoneally with 0 (vehicle), 20, 36, or 62.4 mg/kg mescaline hydrochloride, and after, only a single pairing saccharin consumption was significantly suppressed in all groups injected with mescaline (maximum suppression at 36 mg/kg). In other groups of rats, amphetamine (administered intraperitoneally at 0, 2, 4, and 8 mg/kg) was given following saccharin consumption, and significant aversions were again evident at all doses (maximum suppression at 2 mg/kg). Control subjects consumed at high levels following the saccharin-saline pairing. Subsequent work by Cappell and his colleagues [102] replicated Lester et al. [100] by reporting dose-dependent ethanol-induced CTAs in male Wistar rats and extended the classes of drugs that were effective in inducing aversions to morphine and chlordiazepoxide (3, 6, and 9 mg/kg; intraperitoneal). Importantly, this work revealed that while aversions were dose-dependent, the strength of the aversions and the doses at which significant aversions were evident varied across drugs, suggesting drug-specific aversive effects. Concurrent with (and subsequent to) these initial investigations, a wide range of drugs of abuse known for their ability to support self-administration [103] induced taste aversions as well (see Table 2 for a comprehensive list of various drugs of abuse effective in inducing conditioned taste aversions), suggesting that such drugs produce a number of stimulus effects (both rewarding and aversive).

Almost immediately upon these various demonstrations, a question was raised as to how drugs that were readily self-administered could also be aversive (as indexed by taste aversion learning; see [127, 128], i.e., the two opposing stimulus effects seemed paradoxical. At the outset, it was recognized that these two effects, i.e., rewarding and aversive, were generally assessed via different procedures (and generally in different laboratories). As such, demonstrations of these multiple stimulus effects may be a function of the specific procedure under which they were assessed and not necessarily paradoxical. As examples of these differences, Cappell and his colleagues [127] noted that with work assessing the self-administration of drugs, the drug is generally administered intravenously and under the control of the subject (for a discussion of alternatives, see [10, 129]), whereas in typical taste aversion studies, subjects are given the drug intraperitoneally, subcutaneously, or orally ([34, 130, 131]; though see [132–136] for evidence of taste aversions induced by intravenously delivered drug) and at the control of the experimenter and not the subject (though see [117, 137–139] for demonstrations of aversions induced when the drug was self-administered and/or under the control of the subject).

In addition to these basic procedural differences in drug self-administration vs. taste aversion learning, such demonstrations of the rewarding and aversive effects were often assessed under different parametric conditions, e.g., with different sexes, at different ages, in different strains, at different doses, and under different deprivation schedules, following acute and chronic exposure. The possibility that demonstrations of reward and aversion were a function of simple parametric differences between such demonstrations was soon dismissed with reports that the aversive and rewarding effects of many drugs of abuse could be seen in a design that concurrently assessed these effects which assured that the parametric conditions under which any effects were tested were identical. For example, Wise et al. [137] gave rats access to saccharin and then immediately allowed them to self-administer apomorphine (0.5 mg/kg per infusion; all subjects had previous experience with the intravenous self-administration of amphetamine). On the subsequent exposure to saccharin, 10 of the 11 subjects trained and tested displayed aversions to the apomorphine-associated saccharin solution with the degree of the aversion directly related to the amount of apomorphine self-administered during the initial training session. Thus, both the rewarding (self-administration) and aversive (CTA) effects of apomorphine were evident under the same parametric conditions (and at comparable doses), suggesting multiple (and opposing) stimulus effects of the drug. In a related study, White et al. [140] reported that rats injected with morphine after running down a straight alley to obtain food ran faster to obtain the food (reward) but failed to consume it (aversion), again revealing dual (and concurrent) effects of a drug, in this case morphine. Interestingly, animals given the emetic LiCl under the same conditions displayed reduced running speed to obtain the food and failed to eat the food, as well. In related work, Ettenberg and Geist [138, 139] have reported both positive and negative effects of cocaine in a runway model. In this design, animals are allowed to run down a straight alley for an intravenous injection of cocaine. After several such trials, the latency to leave the start box decreased (indicative of cocaine's rewarding effects) and the running time to enter the goal box increased as animals began to retreat from the goal box with further training (indicative of cocaine's aversive effects). Ettenberg et al. suggested that the immediate actions of cocaine were rewarding (decreasing response latencies) that were quickly followed by an opponent process crash that resulted in an approach/avoidance reaction and increased running time as animals retreated from (avoided) the goal box that was associated with cocaine (see also [141]; for evidence of this time-dependent opponent process of reward/aversions, see [142]).

## 8. Combined Taste Aversion/Place Preference Procedure

Shortly after the demonstrations by Wise et al. [137] and White et al. [140], Reicher and Holman [143] used a different procedure to assess the aversive and rewarding effects of amphetamine. Specifically, this group used a combined conditioned taste aversion and conditioned place preference (CTA/CPP) design in which they gave female Sprague-Dawley rats an intraperitoneal injection of amphetamine (1.43 mg/kg) and placed them on one side of a two-compartment shuttle box during which they had access to a novel-flavored solution (banana or almond). On the next day, the animals were injected with the amphetamine vehicle and placed on the opposite side of the shuttle box with access to the other novel solution (almond or banana). Six such alternating trials were given followed by tests for side and flavor preferences. Under these conditions, amphetamine induced significant taste aversions and place preferences, again demonstrating both aversive and rewarding effects of the same drug and under identical parametric conditions. Subsequent to the initial work by Reicher and Holman, a variety of drugs have now been shown to support both effects in the combined CTA/CPP procedure including 3,4-methylenedioxypyrovalerone (MDPV) [144], *α*-pyrrolidinopentiophenone (*α*-PVP) [104, 145, 146], nicotine [147], amphetamine [148–150], morphine [150–157], cocaine [158–160], alcohol [161], and caffeine [162]; for several drugs, e.g., ethanol [163] and ∆^9^-tetrahydrocannabinol (THC) ([164, 165], both taste and place aversions were reported with the combined design (for reviews, see [166, 167]).

The advantage of using a combined procedure to examine a drug's aversive and rewarding effects in the same animal is that it addresses the concern that the two effects are simply a function of different experimental conditions under which they are tested (see above). While this is true, the combined procedure as generally used does train the animal in a serial manner, i.e., the animal is given access to some novel solution, e.g., saccharin, injected with the drug and then put on one side of the place preference apparatus. Under such conditions, one could argue that acquisition of the CTA itself or the conditions under which the CTA is generally trained and tested, i.e., water deprivation, could impact the acquisition (or display) of the place preference. As such, the measure of reward in terms of place preference conditioning within the combined design might differ from what one would see if place preferences were assessed separately.

Although there are many studies using the combined design (see above), there are only a few that have addressed this potential confound. For example, in one such study, animals were given morphine-induced taste aversion training, and once aversions were established, the same animals were assessed for place preference conditioning with morphine. Place preferences were then compared between groups that had the aversion history vs. those that had been given control injections during the taste aversion training, i.e., control subjects with no pairings of the taste with morphine. Under these conditions, there were no differences between animals with or without the taste aversion history, as morphine-induced place preferences were similar for both groups [153]. These results suggest that having a history in which a specific drug induced an aversion had no effect on its ability to induce a place preference for that same drug. While this addresses the effects of an aversion history on place preference conditioning, it does not address the possibility that the procedures used in the combined design to induce an aversion might impact the acquisition of the place preference. One factor that might impact such learning would be water deprivation (or its associated stress). In the combined design, animals are generally water deprived to encourage consumption, but it is present as well during the place preference assessment, a condition not typically used in independent assessments of place preference conditioning. In a recent study, Dannenhoffer and Spear [147] examined the combined CTA/CPP procedure with nicotine in nondeprived adolescent and adult rats. To induce drinking in these nondeprived animals, a highly palatable sucrose/saccharin solution was given after which the animals were injected with nicotine and placed on one side of a place preference chamber. As expected, nicotine induced significant taste aversions and place preferences, and importantly, place preferences (and taste aversions) were similar to those reported in independent assessments of each. Further, adolescents were more sensitive to the rewarding effects of nicotine (and less sensitive to its aversive effects) relative to adults (for comparison, see [168] who reported these same relative sensitivities of CPP and CTA when separately assessed). Other comparisons across studies have shown that place preference conditioning is comparable when assessed in a combined CTA/CPP design or as an independent CPP and that manipulations in either design impact place preference conditioning similarly (see [152, 157] for assessments of the combined CTA/CPP assay with morphine compared to [169, 170] for assessments of morphine using only CPP; for a similar comparison with MDPV, see [171] compared to [172]; for *α*-PVP, see [104] compared to [173, 174]; and for caffeine, see [162] compared to [175]).

## 9. Implications of the Aversive and Rewarding Effects of Drugs

The fact that drugs have both rewarding and aversive effects raises an interesting issue regarding their possible role in drug intake. Specifically, the balance of these two effects may be important in the likelihood of a drug's initial use and its continued (regulated) intake (see Figure 3). Further, we are suggesting that it is this very balance that predicts the abuse vulnerability of a specific drug [20, 137, 141, 166, 176–179]. If the rewarding effects of the drug (at any given dose) are greater than its aversive effects at that same dose, the abuse vulnerability of this drug might be predicted to be high as intake may increase with its overall greater affective value. If at the outset the drug's aversive effects (at any given dose) exceed its rewarding effects at that same dose, it might be expected that drug intake would not continue and the drug would have limited abuse potential. It is important to note that this balance is not fixed for any specific drug as a wide range of factors have been reported to affect both its rewarding and aversive effects (see below) which, in turn, can shift the affective balance. It is also important to note that the nature of the drug's rewarding effects changes with more frequent and chronic use (from positive associated with acute and regulated intake to negative associated with dysregulated intake and the onset of dependence, anhedonia, and withdrawal (see [4–7]). Although under these latter conditions, drug intake may still be a function of the balance of reward and aversion; the very nature of anhedonia may weaken the relative contribution of the drug's aversive effects as individuals use the drug for relief from withdrawal despite their aversive effects which would normally limit intake.

## 10. Dissociation between the Aversive and Rewarding Effects of Drugs

The fact that these two stimulus effects are evident in the same animals and often under similar parametric conditions supports the position that a drug has multiple affective properties. Interestingly, it appears that these two effects can be dissociated. For example, Verendeev and Riley [150] (see also [180]) have reported that animals trained in a combined CTA/CPP procedure with morphine (5 or 10 mg/kg, intraperitoneal) or amphetamine (3 or 5 mg/kg, intraperitoneal) acquired taste aversions as well as place preferences; however, there was no relationship between the strength of taste aversion and place preference conditioning for either drug. Interestingly, animals that acquired strong morphine-induced taste aversions were just as likely to display weak or strong morphine-induced place preferences. Similarly, animals that acquired weak morphine-induced taste aversions were just as likely to display weak or strong place preferences (for related findings with serial conditioning of CTAs and CPPs, see [180]). That is, there was no relation between the two measures. The same pattern emerged with amphetamine. King et al. [171] have also reported similar independence with the synthetic cathinone, MDPV. In this report, males and females both acquired dose-dependent taste aversions with males displaying greater aversions than females. On the other hand, while both sexes acquired MDPV-induced place preferences, these were independent of sex and correlational analysis between the degree of taste aversions and place preferences did not reveal a consistent relationship between the two measures (see [145] for related findings with the synthetic cathinone a-PVP in which both males and females displayed significant and dose-dependent CTAs (M > F), but only males displayed significant place preferences).

The apparent dissociation of taste aversions and place preferences as measured in the combined CTA/CPP design argues that these two effects occur concurrently but are not related. The fact that the aversive effects of the drug are associated with taste (CTA) while the rewarding effects are associated with a specific place (CPP) is likely a function of the relative selectivity of taste and environment conditioning with these specific affective properties (see [33, 38, 40]; for a review, see [34]). Although apparently dissociable, any attempt to relate these behaviors in a correlational analysis should be made cautiously, given that CTA and CPP procedures may differ in their relative sensitivity as measures of the aversive and rewarding effects of drugs, respectively. For example, CTA may be less sensitive as a measure of the aversive effects of a drug than CPP is as a measure of its rewarding effects, and the drug's aversive effects may not be accurately reflected in the expression of taste aversions. Conversely, CPP may be less sensitive as a measure of the rewarding effects of a drug than CTA is as a measure of its aversive effects. That is, the drug's rewarding effects may not be accurately reflected in the expression of place preferences. As such, any attempt to relate these behaviors in a correlational analysis should be made cautiously. Interestingly, under conditions where taste aversions and place preferences have been analyzed in individual subjects most sensitive to either aversive (high CTA) or rewarding (high CPP) effects of drugs, there still is no consistent relationship between the ability of either drug to produce these effects (see [144, 150]), supporting the ability of the aversive and rewarding effects to cooccur and at the same time being dissociable—a position consistent with the drugs having cooccurring, but unrelated, effects.

Such a position is supported by other assessments of drug-induced taste aversions and place preferences that have found similar dissociations between the two effects in a number of studies evaluating the impact of a variety of manipulations on their acquisition and display, e.g., age [147, 168, 181], sex [145], strain [181–183], drug history [146, 152, 182, 184], drug interactions [116], genetic knockouts/knockins [185, 186], lesions [133, 187], state dependency [188], role of DARRP-32 [189], effects of LPS [190], effects of ^56^Fe particles [191], neuroanatomical and neurochemical mediation [157, 192, 193], and receptor subtype [186, 194]. For these assessments, CTA and CPP were differentially affected, suggesting that the two were unrelated, i.e., if related one would expect that the two effects would be similarly impacted. In the above evaluations, CPP could be seen with no evidence of a CTA (and vice versa) or CPP could be increased and CTA decreased (or vice versa) by chemical and neuroanatomical challenges. Although these demonstrations were generally made with separate analyses of reward and aversion, i.e., using the CTA (or conditioned place aversion) design to assess the drug's aversive effect and the CPP design to assess reward, some were made with the combined design demonstrating again that the dissociations were not a simple function of parametric conditions.

One specific manipulation that deserves special attention is that of dose. As noted in the clinical literature (see above), the rewarding and aversive effects of some drugs were reported to be dose-dependent, specifically rewarding at low doses and aversive at higher ones. While there is evidence of dissociations between place preferences and taste aversions based on studies for which the doses supporting the two effects differ (see [161, 162, 164, 165, 195]), it is important to note that under most of the assessments cited above reporting the dissociation of CTAs and CPPs, comparable doses were administered, yet the two indices of the drug's affective properties were still differentially affected by various manipulations [116, 145–147, 152, 159, 168, 181, 182, 188, 191], i.e., the different effects reported for CTA and CPP were not simply due to animals being tested under different doses in the two designs.

## 11. Nature of the Aversive Effects of Drugs

The present review has discussed conditioned taste aversions in the context of their origins and extensions. As such, it has used the animal's suppression of consumption of a specific taste following its pairing with either a toxin or drug of abuse to be a function of the compound's aversive effects that become conditioned to the taste itself. Noting that drugs of abuse have aversive effects that may limit (or modify) their intake suggests that these effects may be important in regulated drug intake; however, such a position does not indicate their nature which has been somewhat elusive over the history of the phenomenon of taste aversion learning [34]. The present review is somewhat neutral on this issue, but suffice it to say, the literature has had much to discuss (and debate) regarding the basis of taste aversion conditioning. At the outset of work on this phenomenon [33, 196], the avoidance was thought to be a function of conditioning of the radiation-induced gastrointestinal effects, e.g., sickness. The resulting avoidance was a reflection of conditioned sickness/malaise itself, i.e., a conditioned aversion to that taste [38]. As reported by Garcia and Kimeldorf [197], radiation localized to the abdomen induced significant taste aversions at doses that had no effect when targeted to other areas (including the head; higher doses localized to the head, pelvis, or thorax did produce aversions, but even here, they did not approximate those targeting the abdomen). Garcia and Kimeldorf noted that abdomen radiation induced aversions at the same dose that decreased gastric distension and transit, leading them to conclude that gastric disruption is the stimulus likely necessary to condition aversions. As other agents (mostly toxins) were reported to induce aversions, it was assumed that these compounds also produced sickness or malaise, but these conclusions were generally made in the absence of direct corroborative evidence of such effects (and often in the context of contrary evidence, e.g., the general inability of antiemetic drugs to affect CTAs [198, 199], the ability of antiemetics to induce CTAs themselves [109, 200], and the absence of a relationship between the degree of sickness and CTAs [201].

A similar explanation was used by many to account for the avoidance of taste paired with drugs of abuse which, in part, created the initial paradox of how drugs of abuse could be both aversive (via sickness) and rewarding at the same time. While conditioned aversions (sickness) were often applied to the suppression of consumption of tastes paired with drugs of abuse, others challenged this position. For example, in an elegant series of studies, Parker assessed taste reactivity as an index of the sickness-inducing effects of drugs and found that although most drugs of abuse resulted in the suppression of consumption of solutions paired with the drug (see [202]; see also above; Table 2), these same drugs did not produce signs of sickness in the taste reactivity assessments ([203]; for recent work with LiCl vs. lactose, see [204]). In assessments of taste reactivity, a taste previously associated with some drug, e.g., LiCl, amphetamine, and cocaine, is infused into the animal's mouth via an indwelling cannula and both aversive and positive taste reactions to the infused solution are recorded. If the taste has been paired with LiCl (and other emetics), a host of aversive taste reactions are increased, e.g., gaping, chin wipes, and paw treading, which are used as an index of sickness/malaise induced by the conditioned taste (via its pairing with a drug that induced such effects unconditionally; see [205, 206]). As noted, tastes paired with drugs of abuse generally do not induce aversive taste reactivity (for reviews, see [207–209]). Parker and her colleagues concluded from these analyses that drugs of abuse do not induce sickness (as indexed by the taste reactivity test), and thus, the suppression of consumption of the taste associated with such drugs is not a function of a conditioned aversion to the taste itself. Importantly, Parker has shown that even drugs such as LiCl which do induce aversive taste reactivity (reflective of conditioned sickness) do not suppress the intake of LiCl-associated solutions through this mechanism in that antiemetics can attenuate aversive taste reactivity while leaving LiCl-taste aversions intact [210] (for a review, see [199]). From her analysis of the basis of the suppressed consumption of solutions induced by drugs of abuse, Parker suggests that sickness plays no role and even questions the role of sickness in suppression induced by emetics such as LiCl (for evidence critical of Parker's position of the importance of sickness in taste aversion learning using measures other than taste reactivity, i.e., lick pattern and rate, to assess sickness and palatability shifts, see [211–215]; see also [216, 217]).

Given the diminishing role of sickness as the common mediator of the effects induced by various agents to induce taste aversions, others turned to different mediators of such effects. In this context, it was generally stated that aversion-inducing agents had toxic (adverse) effects (but not necessarily sickness or malaise) that were responsible for taste aversion conditioning [31]. As such, interpretations became couched not in sickness but in rather general terms of toxicity. Such a general term conveyed no clear mechanisms of the toxicity, and, further, drugs with reported toxicity in other behavioral toxicological screens did not always induce aversions [41] (for a discussion, see [31]). Also, when drugs of abuse were reported to induce taste aversions (see above), the explanations were even more difficult in the context of general toxicity as such drugs in addition to being rewarding in other preparations produced no obvious toxic effects at the doses tested [128] (see [20]). To address this issue, a number of individuals noted that such drugs of abuse were aversive by disrupting normal homeostasis [31, 127, 128, 207, 214]. That is, given that general homeostasis is a well-defended state (see [128]; for related discussion on drugs of abuse in terms of their transition from use to abuse, see [5]); any disruption in this state is perceived as dangerous and defended. In one of the first reports on this possibility, Gamzu [128] discussed drug novelty itself as being the necessary condition for disruptions of homeostasis and in conditioning taste aversions (see [218] for a related position that argued that the actual rewarding effects of drugs were the novel stimulus that induced taste aversions). Although drug novelty is important in the conditioning of taste aversions (as exposure to the drug prior to conditioning weakens the acquisition of taste aversions), several arguments challenged this specific account. For example, as noted above, a number of classic toxins such as strychnine and cyanide as well as convulsants fail to induce CTAs (see [41]). It is difficult to explain how drugs with clear toxicity fail to induce a novel state. More importantly, although drug history weakens taste aversion acquisition, with repeated conditioning trials (where the taste and familiar drug are repeatedly paired), aversions do develop despite the fact that the drug is no longer novel (for a review, see [219]).

Disruptions in homeostasis can be produced by toxins, chemicals with adverse effects, and drugs of abuse, and according to the evolutionary importance of recognizing such disruptions as potentially dangerous, all such compounds should be effective in inducing taste aversions (and for the most part they are). However, stating that such disruptions are important in inducing aversions does not suggest that there is a common mechanism mediating all of these compounds. For example, even though drugs of abuse are rewarding as assessed in standard operant and Pavlovian designs that index these effects, collateral effects such as sickness (morphine), hyperthermia (synthetic cathinones [145]), anxiety (cocaine and amphetamine [138, 139]), sedation (barbiturates), hypothermia (alcohol [220]), and opponent process-related withdrawal (cocaine and morphine [136, 183, 221–223]), may be the stimuli important in inducing aversions by virtue of their ability to disrupt homeostasis. What is critical about this explanation of homeostasis is that the aversive effects of drugs that condition aversions are drug (and parameter)-specific (and not due to a general issue of malaise or stress; for a discussion of a potential common mediator, i.e., fear, see [224]). It is important to note here that few of the proposed mediating stimulus effects have been directly tested and the failure of specific toxins to induce aversions still needs to be explained (see [31] for an explanation of failure of several rodenticides and toxins). Further, over the past 20 years, a wide range of neuroactive compounds as well as neurochemicals involved in the modulation of normal neuronal function (and behaviorally active) are not effective in inducing CTAs, failures that challenge a simple homeostatic disruption as mediating aversion learning, e.g., interleukin-1B [225], interleukin-6 [226], leptin [227], GHR-R antagonist JMV 2959 [228, 229], L-tryptophan [230], N-acylphosphatidylethanolamine [231], and oleoylethanolamide [232].

Although each of these mechanistic accounts has been offered as a basis for taste aversion learning and most papers refer to one of these interpretations in their analysis of CTAs, no individual perspective is generally accepted. Independent of which interpretation eventually garners consensus, all argue that the drug (whether a toxin, exogenous chemical agent, peptide, neurochemical, or drug of abuse) has some adverse effect that induces aversions (for an alternative interpretation that argues that the avoidance of drug-paired tastes is a function of a reward comparison in which the taste is devalued relative to the injected drug, i.e., anticipatory contrast, see [155–157, 233–235]; see [20] for a review of the reward comparison hypothesis).

## 12. Implications for the Aversive and Rewarding Effects of Drugs to Use and Abuse

The fact that drugs of abuse have both aversive and rewarding effects is now well characterized by a wide range of such compounds. The fact that the two effects are also dissociable is important given that they can be differentially impacted by a host of parametric, experiential, and subject factors (see above). That is, the balance between these two affective properties can be differentially impacted by these factors and, in turn, can change abuse vulnerability. In this context, the hypothetical interaction of aversion and reward as illustrated in Figure 3 is not static but is one that will differ depending upon the drug examined (including its dose, route of administration, and frequency of use) and the myriad of subject (sex, age, and genetics) and experiential (drug interactions, drug history, drug expectancy, and conditioning history) factors that can modulate each affective response (for a discussion, see [166, 176, 236]). Knowing the impact of these factors on drug aversion and reward and their balance should provide insight into the drug's use and its abuse vulnerability.

The questions then become how this impact occurs and under what conditions. The complexity of these questions becomes clear when one examines facets of drug-taking (see [4]) that range from controlled to dysregulated use (abuse). In this context, aversion and reward (and their balance) could impact the likelihood of initial drug intake and its maintenance as well as the dysregulation of drug intake that may escalate to abuse. Although each of these is important in assessing how drug use and abuse may be impacted by the affective properties of drugs, relatively little has addressed these specific issues. This review will highlight some of the work in these areas and what could be done.

These issues have recently been addressed by De Wit and Phillips [13] in their review “Do initial responses to drugs predict future drug use?.” In this review, they raise the point that drugs can vary on a number of characteristics, including the magnitude, quality, and duration of their effects, all of which may impact subsequent use. One characteristic which is highlighted in their review is the affective valence of a drug's effects, i.e., the positive and negative effects that may facilitate and discourage use, respectively (similar to the affective properties noted in the present review). Using both retrospective and prospective assessments (along with human laboratory studies), they then assess for a variety of drugs (alcohol, nicotine, caffeine, psychostimulants, heroin, and marijuana) whether the initial response to these compounds is associated with subsequent use and/or abuse. As they describe, individuals differ significantly in their initial response to these drugs (as a function of environmental and genetic influences) and that for several drugs the initial responses (either positive or negative) are correlated with subsequent use (and in some instances substance use disorder). For example, with alcohol, individuals who initially display greater stimulant-like effects as breath alcohol concentrations are rising (see [237]) and feel fewer depressant effects as these levels decrease [238] are more likely to use and abuse alcohol. Conversely, those individuals that experience unpleasant effects are less likely to subsequently consume alcohol, effects and outcomes similar to what was previously described for individuals with metabolic differences in the ability to metabolize the alcohol metabolite acetaldehyde (see above; see also [22, 239]).

For other drugs (e.g., nicotine), the initial positive response was a better predictor of use and abuse (although negative responses limited intake under some conditions). For others (e.g., marijuana), only initial positive responses were associated with later use that, in turn, had little association with initial negative reactivity. For caffeine, unpleasant effects or negative subjective responses predicted lower consumption. Finally, for heroin, individuals having greater positive experience were more associated with later abuse (although no data have been reported on the relative association with any negative effects, e.g., nausea). In a summary of their work, De Wit and Phillips [13] cautioned that an understanding of the contribution of the initial affective response to a drug to its later use and/or abuse must be assessed in the context of many other factors such as expectancies, cognitive control, drug history, learning, and physical dependence, all of which clearly impact the likelihood of continued drug use and its escalation (e.g., the fact that individuals adjust doses of heroin or become tolerant to its aversive effects may limit generalization about the relative role of initial positive and negative effects to its continued use).

Interestingly, De Wit and Phillips [13] also assessed related work on positive and negative drug effects in animal models and noted the relative paucity of data assessing affective valence in nonhuman subjects and its relationship to drug intake in animals. The one area for which considerable data have been reported has used selectively bred animals (lines selectively bred for specific phenotypes) and inbred animal strains (derived from full-sibling mating that maximize genetic homogeneity) as their focus (for reviews, see [176, 236, 240]). The creation of selectively bred lines that are differentially sensitive to the aversive effects of drugs has been reported for many years (see [241, 242]). Such animals (taste aversion prone and taste aversion resistant, TAP and TAR, respectively) display significant differences in their ability to acquire aversions induced by a variety of drugs, e.g., cyclophosphamide, LiCl, and emetine hydrochloride [241, 242], and importantly by drugs of abuse, e.g., alcohol ([243]; see also [244]), with the TAP animals displaying aversions at lower doses and acquiring aversions at a faster rate than the TAR animals. These differences in aversion learning do not reflect differential abilities to learn in general as TAP and TAR rats are similar in other learning preparations that do not utilize aversion conditioning (see [245, 246]).

Although Elkins and his group did not assess the potential contribution of these differential sensitivities of the aversive effects of alcohol (and cocaine) to drug intake in these same animals, others have done related work and have shown in both inbred strains and other selected lines that animals that show greater drug-induced taste aversions induced by specific compounds such as alcohol, methamphetamine, and heroin are less likely to self-administer those same compounds (orally or intravenously) (see [166, 176, 236]). For example, the Wistar Kyoto (WKY) rat strain that generally displays low consumption of alcohol in free-choice assessments displays strong taste aversions to novel solutions paired with exogenously administered ethanol (and differ significantly in both measures relative to the Marshal strain (M520) that generally consumes high levels of alcohol and only weak aversions to ethanol-paired solutions). In other words, there is an inverse relationship between alcohol consumption and its aversive effects (see [247, 248] for similar comparisons between the high alcohol-consuming Wistar Kyoto hyperactive rat (WKHA) and the WKY and spontaneously hypertensive rat strains).

The vast majority of work assessing the relationship between the aversive effects of drugs and drug intake has been with inbred strains of mice, specifically the C57BL/6J and DBA/2J strains. These two strains have been examined for alcohol preference and ethanol-induced taste aversions in a number of contexts and have consistently been shown to display an inverse relationship between alcohol intake and ethanol-induced taste aversions. Specifically, DBA mice (alcohol avoiding) acquire ethanol-induced taste aversions at a lower dose/concentration and at a faster rate relative to alcohol-preferring C57 mice. In a comprehensive analysis of 15 inbred mouse strains, Broadbent et al. [249] reported a significant inverse relationship between alcohol consumption and ethanol-induced taste aversions, suggesting that the sensitivity to the aversive effects of alcohol may serve as a protection against elevated alcohol intake (see [250] for a similar inverse relationship between oral alcohol intake and ethanol-induced place aversion conditioning, another index of the aversive effects of drugs; see [251] for related work showing that ethanol-induced place preference conditioning was not significantly correlated with alcohol consumption, suggesting a greater role for the aversive effects of alcohol in strain differences in alcohol acceptability).

Other work has focused on selective breeding to assess the relationships between the aversive effects of drugs and their self-administration. For example, Phillips and her colleagues have reported similar findings with methamphetamine. Specifically, rats that are selectively bred for high oral self-administration of methamphetamine were less likely to display methamphetamine-taste aversion (an index of its aversive effects) and more likely to display methamphetamine-place preferences (an index of its rewarding effects) than rats selectively bred for low methamphetamine intake (see [183]; see also [252, 253]). Interestingly, rats selectively bred for low and high drinking of methamphetamine displayed no differential aversive (as measured by CTA) or rewarding (as measured by CPP) effects of cocaine, showing that the genetic sensitivity to the aversive and rewarding effects of methamphetamine does not impact cocaine susceptibility [195]. Such findings of the inverse relationship between the aversive effects of a drug and its tendency to be self-administered in selectively bred strains are not limited to methamphetamine and the low and high drinking mice. For example, our laboratory has also focused on this issue in selectively bred rat strains, specifically the Lewis (LEW) and Fischer (F344) strains that are well characterized for their differences in intravenous self-administration of a variety of drugs. These two strains were originally selectively bred for cancer susceptibility and tissue inflammation (for discussion of the origins of these lines, see [176]) but subsequently were shown to differ for a myriad of other behaviors, including stress reactivity and drug intake, although the two strains were not selectively bred for differences in these latter two effects. In relation to drug intake, the LEW and F344 rat strains are well characterized for their differences in the self-administration of a variety of drugs of abuse, including alcohol (oral), morphine, etonitazene, methamphetamine, cocaine, and nicotine, and under most comparisons, LEW rats self-administer greater amounts of drugs than does the F344 strain (for a review, see [176]). The general conclusion regarding these genetic differences in drug intake is that the two strains differ significantly in their sensitivity to the drugs' rewarding effects, a conclusion supported by the fact that for a variety of drugs the LEW strain displays conditioned place preferences at lower doses than the F344 strain (see [176]). Interestingly, however, these strains also differ significantly in the aversive effects of the same drugs. For example, we have demonstrated for morphine [254–256], alcohol [163], and nicotine [257] that the F344 strain acquires morphine-, alcohol-, and nicotine-induced taste aversions at lower doses than the LEW strain. Such differences in sensitivity to the aversive effects of these drugs are not a general function of learning as these strains differ in the opposite direction for the drugs' rewarding effects as indexed by place preference conditioning (L > F). Further, the two strains do not differ in aversions induced by compounds with no abuse potential, e.g., the emetic LiCl [258], the kappa opiate receptor agonist U50,488H [255], the delta opiate receptor agonist SNC80 [255], and the peripherally acting mu opiate receptor agonist loperamide [256].

Thus, similar to work with inbred strains, we see an inverse relationship between drug intake and the relative sensitivity to taste aversion conditioning, i.e., animals readily self-administering the drug display weaker taste aversions (and vice versa), again substantiating a genetic component mediating the basis for drug use. In that context, there are several important caveats. First, when cocaine is used as the aversion-inducing agent, the LEW strain displays greater aversions, i.e., the LEW strain self-administers cocaine at higher rates than the F344 strain and displays greater cocaine-induced taste aversions [259] (see [260] for related findings with caffeine). While this challenges the inverse relationship reported with alcohol, morphine, and nicotine, it should be noted that such a finding is not necessarily inconsistent with the position that drug intake is a balance of reward and aversion. In the case of cocaine, the LEW strain is more sensitive to both affective properties, but the balance may nonetheless be shifted toward reward, supporting greater self-administration (see above discussion on the balance of reward and aversion). A second caveat concerns the implications of the findings in general for a genetic mediation of the aversive and rewarding effects of drugs based on the selective breeding model. While the difference between the LEW and F344 rat strains clearly represents effects that have genetic influence, it does not mean that these differences cannot be impacted by environmental factors. Support for this position comes from work on cross-fostering in the strains. For example, we have reported that while LEW and F344 stains differ in their sensitivity to the aversive effects of morphine (F > L; see [254]), these differential sensitivities are partially reversed with cross-fostering. That is, F344 animals that normally display robust morphine-induced aversions resemble pups for the LEW strain that are relatively insensitive to morphine if they are reared by a LEW dam; conversely, LEW animals that generally show weak morphine-induced aversions acquire strong aversions (similar to the F344 strain) if reared by a F344 dam [261]. Partial reversals were also seen when cocaine was used as the aversion-inducing drug, i.e., the F344 strain that normally displays weak cocaine-induced taste aversion display strong aversion characteristics of the LEW strain if reared by a LEW dam (see [176]; for reports of reversals of other behavioral effects by cross-fostering, see [262, 263]).

The major work showing how the aversive (and rewarding) effects of drugs may impact drug intake has primarily been within various genetic models (see above; for related work with KO mice, see also [186, 189, 264–266]; see also [267, 268] for effects of aldehyde dehydrogenase type 2 KO and alcohol consumption and acetaldehyde brain, blood, and liver levels). It is important to note here that the aversive effects of drugs are impacted by a variety of other factors such as sex [177], drug history [219], and age [269, 270], and the impact of these factors on drug use and abuse has only recently been explored in this context. It will be critical in such analyses that the impact of their effects be explored not only on the initial use of various drugs of abuse (i.e., reflecting the drug's initial acceptability) but also on how these factors impact the likelihood of drug escalation and choice as well as relapse of extinguished drug response (reinstatement) (for an example of such assessments on the complexity of drug-taking, see [271]).

## 13. Drug Regulation

Although the aversive effects of a drug on its subsequent intake have primarily been discussed as a limiting or protecting factor (see [20, 141, 236]), these effects may also be important to the regulation of normal intake or dysregulation of intake that transitions drug use to drug abuse. This possibility has recently been suggested by our laboratory in discussions on the role of drug states in regulated drug intake [272, 273]. A principal feature of drug addiction is overconsumption followed by a reduced ability to control the desire to obtain drugs regardless of the risks involved, ultimately resulting in compulsive drug seeking [7]. The possibility that environmental stimuli associated with the postingestive rewarding effects of drugs strongly motivate consumption has guided much of the research exploring the role of neuroadaptations in the mesolimbic and mesocortical dopamine systems as well as in the prefrontal and orbitofrontal cortices mediating responses to drug rewards [5, 274]. There is little doubt that the memory of highly rewarding postingestive drug effects can strongly influence expectations about the outcomes a particular drug will produce. The strength to which drug-related contexts (e.g., time and space) can excite retrieval of those memories is a key determinant of current and future consummatory behavior [275, 276].

However, the response to drug-related cues involves more than excitatory associations that predict rewarding postingestive outcomes that, in turn, generate drug-taking. As demonstrated by the majority of individuals consuming drugs, the patterns of drug intake are generally well regulated, indicating that the capacity for drug-related cues to evoke intake is not without limits [277, 278]. That is, bouts of drug intake stop even when environmental cues (and the drug itself) that have gained the power to initiate intake are still present. Such regulatory control involves higher-level learning and memory processes that counter the power of palatable drugs (and drug-related stimuli) to inhibit further intake [271, 279–281]. The same environmental stimuli associated with the rewarding consequences on some occasions, e.g., at the outset of consumption, can also predict nonrewarding or even aversive consequences on other occasions, e.g., toward the end of a bout of drug use. Thus, both excitatory and inhibitory associations are formed between drug cues and positive and negative postingestive outcomes, respectively, depending on the context. The ambiguous nature of the associations between drug-related cues and these consequences suggests that additional signals must be used to predict when taking the drug will produce rewarding outcomes and when the drug will produce nonrewarding or even aversive effects, leading to an end in the bout of drug intake. We are suggesting that regulatory control of drug intake is dependent in part on the ability of contextual drug states to disambiguate conflicting associations between drug cues and postingestion outcomes. In this framework, although the initiation of drug-taking depends on the activation of excitatory associations that predict rewarding effects, contextual stimuli suppress intake by activating the inhibitory associations between the same drug cues associated with nonrewarding or aversive postingestive outcomes. Dysregulated intake, in turn, may be a function of poor control by these drug state cues that would produce an imbalance that favors the excitatory associations, leading to overconsumption (see evidence by [282–284] for the role of similar processes involved in the regulation/dysregulation of food intake).

Although the processes of cognitive inhibition described above have primarily been implicated in the regulation of food intake, the imbalance between inhibitory and excitatory control mechanisms may also explain why some people progress from regulated to dysregulated drug use. Given free drug access, animals learn to regulate drug intake to achieve a particular level of intoxication by titrating drug levels within the brain and bloodstream [15]. Characteristics of maintained drug self-administration indicate that drug or drug-associated stimuli encountered by an animal in a drug-free state will initiate drug intake, but when the drug level reaches above a satiety threshold, i.e., the minimal drug level at which self-administration is maintained, animals temporarily suspend drug seeking [15, 280]. Consistent with this position, the presence or absence of a drug in the biological system has been demonstrated to serve discriminative functions that signal the availability of certain reinforcers, e.g., food and water [285–288]. Not only can drugs serve as discriminative stimuli in general but also the discriminative control of the training drug can also be generalized to drugs with comparable mechanisms of action [289–292].

We [293] and others [294–297] have extended the analysis on drug discrimination learning to show that interoceptive drug cues can also signal the presence and absence of an aversive outcome using a modified conditioned taste aversion design (for a review of the conditioned taste aversion baseline of drug discrimination learning, see [272]). In one demonstration, rats received PCP followed by a pairing of saccharin with the emetic LiCl on the conditioning day, and on the subsequent 3 days, the same animals received the PCP vehicle followed by paring of saccharin with the LiCl vehicle. Over multiple trials, animals avoided consuming saccharin when it was preceded by PCP and consumed saccharin when it was preceded by the PCP vehicle. The control group that received the same PCP/vehicle injections prior to saccharin, but never the postsaccharin injection of LiCl, consumed high levels of saccharin throughout the study, indicating that the suppressed saccharin consumption in the LiCl-treated group was a function of PCP signalling the saccharin-LiCl contingency rather than an unconditioned suppression on saccharin consumption [293] (for related work with morphine, see [295, 297]).

To date, accumulating evidence that a wide range of drugs can serve such a discriminative function provides clear support for the ability of drug stimuli to modulate consummatory behavior by signalling postingestive outcomes. Similar to the function of satiety cues in food intake regulation, discriminative learning may be important in regulating drug intake. Humans and other animals might use interoceptive drug signals to determine when a sufficient drug level has been achieved and whether to continue or refrain from continued or elevated consumption (see [13] for a discussion of the possible role of the inability to detect such stimulus effects in alcoholics). Such an evaluation of drugs and consequences of intake is governed by prior learning of various consequences of drug use. Further, memory processes represent associations between drug-taking contexts, drug cues, and the consequences of drug-taking acquired over a repeated experience that strongly influence the cognitive inhibition of drug intake. A rich literature has demonstrated that the hippocampus modulates the capacity of any contextual or discrete cues to activate inhibitory associations to suppress the retrieval of memories of rewarding outcomes [298–300]. Hippocampal damage has been shown to impair the ability of humans [301–303] and rats [304, 305] to discriminate interoceptive satiety cues from hunger and to suppress food-reinforced conditioned response overconsumption. Rats with impaired hippocampal-dependent inhibitory control showed greater intake and meal frequency within a shorter interval [306–308] and greater weight gain within weeks [309] or months [310].

Specific to the issue of drug intake, we suggest that neuroadaptations resulting from chronic drug use disrupt the ability of the hippocampus to mediate inhibitory control over responses to drug-related cues. In this context, hippocampal impairments have been implicated to modulate the transition from regulated to dysregulated drug intake. In chronic drug users, various drugs of abuse have been reported to impair the functional integrity of the hippocampus and interfere with learning and memory [311, 312]. Hippocampal lesions have also been demonstrated to increase the oral consumption of alcohol and the intravenous self-administration of cocaine, methamphetamine, morphine, and nicotine in rodents [313–316]. Furthermore, we have recently reported that chronic administration of cocaine interfered with the ability of rats to solve a hippocampal-dependent discriminative task known as the serial feature negative (sFN) discrimination that requires the animals to use contextual signals to disambiguate postingestive outcomes [317]. Interestingly, chronic administration of cocaine in the same animals had no effect on simple discrimination problem that does not require a functional hippocampus, indicating that the type of learning and memory processes required to resolve approach-avoidance conflict in the sFN discrimination task does not rely on nonspecific factors (e.g., motivation and attention) but a higher-level regulatory mechanism dependent on the hippocampus to disambiguate conflicting associations.

Taken together, these data highlight the fact that the hippocampus is critically involved in regulating consummatory behaviors and that chronic drug use uniquely targets hippocampal-dependent forms of learning and memories. If chronic drug use disrupts the hippocampal function to modulate the ability of interoceptive cues of drug satiety to engage inhibitory associations, then chronic drug exposure might reduce the power of drug satiety cues to inhibit intake. In support of this idea, future studies in drug addiction should not be limited to reward- and motivation-based models; rather, future research should also explore a model predicated upon hippocampal functioning underlying regulated drug use that could potentially contribute to preventing the transition to dysregulated drug use and pathological state of drug abuse.

## 14. Conclusions

In this review, we have discussed drug use and abuse in the context of a reward model and have qualified this analysis by arguing that drugs of abuse have multiple stimulus properties (both rewarding and aversive) that need to be considered in any account of drug-taking behavior. We provided evidence that drugs have aversive effects (from both clinical and preclinical populations) and have introduced and discussed these effects in their historical context (generated by work on conditioned taste aversions). We indicate that the aversive effects can occur concurrent with rewarding ones in the same subject trained and tested under identical conditions and that their relative balance is important to the use and/or abuse of the drug. While both rewarding and aversive effects occur, we describe reports indicating that these effects appear dissociable, suggesting that manipulations can impact them differently. We further suggest that an awareness of each affective property and the multiple parametric, experiential, and subject factors that impact them and their relative balance will give insight into use and abuse vulnerability (for example, see [177]). Data supporting such a position were provided by an overview of the relationship between initial and subsequent drug use (in humans) and a more detailed analysis of the inverse relationship between perceived aversive effects of drugs and their intake. We close our review by noting that the interaction of reward and aversion may also be involved within bouts of drug intake as the ability to use the drug state itself to set the occasion for aversive effects that may accompany elevated use. We conclude from these issues that examining a drug's aversive effects (in addition to the myriad of other stimulus effects produced) is critical to understanding drug intake and developing prevention and treatment strategies associated with the transition from use to abuse.

## Figures and Tables

**Figure 1:** Transition from the impulsive (acute) to the compulsive (abuse) patterns of drug-taking. Adapted from Meyer and Quenzer [8] using BioRender.com.

**Figure 2:** Median saccharin preference scores for animals previously given saccharin access during radiation exposure. Redrawn from Garcia et al. [33].

**Figure 3:** A hypothetical model of the aversive and rewarding effects of a drug and their potential interaction to impact its self-administration (which is a function of the overall affective response to the drug). The drug produces both aversive and rewarding effects in a dose-dependent manner. As illustrated in this specific example, the drug's rewarding effects are produced at lower doses that increase the drug's overall affective property that, in turn, drives the drug's intake. With increases in the dose, the drug's rewarding effects asymptote while the drug's aversive effects increase, reducing the overall affective value of the drug and decreasing the drug's self-administration. In this model, the drug's rewarding effects are assumed to initiate and maintain drug intake (at least under acute conditions) while its aversive effects limit it. The nature of such an interaction is not static and depends upon a host of factors (see Sections 11 and 12). Further, the relative contributions of the aversive effects in limiting intake change as drug intake go from regulated to dysregulated given the change in the reward valence from positive to negative. Created with BioRender.com.

**Table 1:** Compounds with adverse or toxic effects effective in producing CTAs.

Compound	Reference
*α*-Naphthylthiourea (rodenticide)	Rzóska, 1954a [32]
1,1,2-Trichloroethane (carcinogen)	Kallman et al., 1983 [44]
1,2-Dicholoethane (probable carcinogen)	Kallman et al., 1983 [44]
1,2-Dichloroethylene (health hazard)	Kallman et al., 1983 [44]
2,3,5-Trimethylphenyl methyl carbamate (neurotoxin)	Nicolaus, 1987 [45]
2,4,5-Trichlorophenoxyacetic acid (herbicide)	Sjödén and Archer, 1977 [46]
6-Formylindolo (3,2-b) carbazole (FICZ) (carcinogen)	Mahiout and Pohjanvirta, 2016 [47]
Acetaldehyde (primary metabolite of ethanol)	Brown et al., 1978 [48]
Acetoxycycloheximide (protein synthesis inhibitor)	Ungerer et al., 1975 [49]
Acrylamide (neurotoxin)	Anderson et al., 1982 [50]
Adriamycin (gastrointestinal tract toxin)	Bernstein et al., 1980 [51]
Aflatoxin B1 (toxic to liver and kidney)	Rappold et al., 1984 [52]
Alloxan monohydrate (diabetogenic agent)	Brookshire et al., 1972 [53]
Arsenic (rodenticide)	Rzóska, 1954a [32]
Atrazine (chlorotriazine herbicide)	Hotchkiss et al., 2012 [54]
barium carbonate (rodenticide)	Rzóska, 1954a [32]
Baygon (insecticide)	Ebeling, 1969 [55]
Benzo[*α*]pyrene (BaP) (dioxins)	Mahiout and Pohjanvirta, 2016 [47]
Boric acid (pesticide)	Ebeling, 1969 [55]
Bufotoxin (neurotoxin)	Ward-Fear et al., 2016 [56]
Cadmium (toxic metal)	Wellman et al., 1984 [57]
Carbaryl (insecticide)	MacPhail and Leander, 1980 [58]
Chloral hydrate (potent sedative)	Kallman et al., 1983 [44]
Chlordimeform (insecticide)	Landauer et al., 1984 [59]
Cisplatin (cytotoxin)	Revusky and Reilly, 1989 [60]
Clorgyline (neurotoxin)	Buresová and Bures, 1987 [61]
Cobalt chloride (toxic to organs)	Wellman et al., 1984 [57]
Cobra venom (neurotoxin)	Islam, 1980 [62]
Copper sulfate (pesticide)	Nachman and Hartley, 1975 [41]
Cyanide (cytotoxin)	O'Connor and Matthews, 1995 [63]
Cycloheximide (protein synthesis inhibitor)	Booth and Simson, 1973 [64]
Cyclophosphamide (gastrointestinal tract toxin)	Dragoin et al., 1971 [65]
Cytoxan (cytotoxin)	Bernstein et al., 1980 [51]
Dactinomycin (cytotoxin)	Revusky and Martin, 1988 [66]
Denatonium benzoate (rodenticide)	El Hani et al., 1998 [67]
Doxorubicin (cytotoxin)	Revusky and Martin, 1988 [66]
Emetine hydrochloride (emetic)	Cannon and Baker, 1981 [68]
Ferric nitrilotriacetate (Fe-NTA) (renal carcinogen)	Irie et al., 2000 [69]
Formalin (systemic poison)	Stricker and Wilson,1970 [70]
Ipecacuanha (emetic)	Rudd et al., 1998 [71]
Krait venom (neurotoxin)	Islam, 1980 [62]
Lead (toxic metal)	Leander and Gau, 1980 [72]
Lipopolysaccharide (endotoxin)	Exton et al., 1995 [73]
Mechlorethamine (vesicant)	Revusky and Martin, 1988 [66]
Mercuric chloride (cumulative poison)	Klein et al., 1974 [74]
Methyl bromide vapor (cumulative poison)	Miyagawa, 1982 [75]
Methylmercury (neurotoxin)	Levine, 1978 [76]
Methiocarb (pesticide)	Mason and Reidinger, 1982 [77]
Metrazol (convulsant)	Millner and Palfai, 1975 [78]
Mesurol (pesticide)	Gustavson et al., 1982 [79]
Sodium fluoroacetate (rodenticide)	Nachman and Hartley, 1975 [41]
n-Butyraldoxime (aldehyde dehydrogenase inhibitor)	Nachman et al., 1970 [80]
N-N-Ethyl-2-bromobenzylamine (neurotoxin)	Archer et al., 1983 [81]
Ochratoxin (mycotoxin)	Clark and Wellman, 1989 [82]
Ozone (toxic to lung)	MacPhail and Peele, 1992 [83]
Paraquat (herbicide)	Dey et al., 1987 [84]
p-Chlorophenylalanine (neurotoxin)	Nachman et al., 1970 [80]
Phenylthiocarbamide (neurotoxin)	St. John et al., 2005 [85]
Picrotoxin (GABA receptor inhibitor)	Chester and Cunningham, 1999 [86]
Red squill (rodenticide)	Rzóska, 1954a [32]
Sarin (neurotoxin)	Landauer and Romano, 1984 [87]
Scorpion venom (neurotoxin)	Islam, 1980 [62]
Sodium cyanide (rodenticide)	Nachman and Hartley, 1975 [41]
Soman (neurotoxin)	Romano et al., 1985 [88]
Staphylococcal enterotoxin B (exotoxin)	Kusnecov et al., 1999 [89]
Strychnine sulfate (rodenticide)	Howard et al., 1968 [90]
T-2 toxin (mycotoxin)	Wellman et al., 1989 [91]
Thallium sulfate (rodenticide)	Nachman and Hartley, 1975 [41]
Thiabendazole (pesticide)	Gustavson et al., 1983 [92]
Thiram (fungicide)	Tobajas et al., 2019 [93]
Tumour necrosis factor *α* (cytokines)	Goehler et al., 1995 [94]
Trichloroethylene (carcinogen)	Kallman et al., 1983 [44]
Trichloromethane (neurotoxin)	Balster and Borsellca, 1982 [95]
Triethyltin (neurotoxin)	MacPhail, 1982 [42]
Trimethyltin (neurotoxin)	MacPhail, 1982 [42]
Triphenyltin (fungicide)	MacPhail and Peele, 1992 [83]
Toluene (systemic toxin)	Miyagawa et al., 1984 [96]
Viper venom (hemotoxic)	Islam et al., 1982 [62]
Vomitoxin (mycotoxin)	Clark et al., 1987 [97]
Xylene (systemic toxin)	MacPhail and Peele, 1992 [83]
Ziram (fungicide)	Baker et al., 2005 [98]

**Table 2:** Drugs of abuse that are effective in producing a CTA. Each drug has the reference for one of the initial studies examining that specific drug.

Compound	Reference
*α*-Pyrrolidinopentiophenone (*α*-PVP) (synthetic cathinone; CNS stimulant)	Nelson et al., 2017 [104]
∆^9^-Tetrahydrocannabinol (∆^9^-THC) (cannabinoid)	Elsmore and Fletcher, 1972 [105]
3,4-Methylenedioxymethamphetamine (MDMA) (hallucinogen)	Lin et al., 1993 [106]
3,4-Methylenedioxypyrovalerone (MDPV) (synthetic cathinone; CNS stimulant)	King et al., 2014 [107]
Amobarbital (CNS depressant)	Vogel and Nathan, 1975 [108]
Amphetamine (CNS stimulant)	Berger, 1972 [109]
Barbital (CNS depressant)	Jolicoeur et al., 1977 [110]
Caffeine (CNS stimulant)	Dickens and Trethowan, 1971 [111]
Cathinone (CNS stimulant)	Goudie and Newton, 1985 [112]
Cannabidiol (CBD) (cannabinoid)	Corcoran et al., 1974 [113]
Cannabigerol (CBG) (cannabinoid)	Corcoran et al., 1974 [113]
Cocaine (CNS stimulant)	Goudie et al., 1978 [114]
CP 55,940 (synthetic cannabinoid)	McGregor et al., 1996 [115]
d-Amphetamine (CNS stimulant)	Cappell and LeBlanc, 1971 [101]
Diazepam (CNS depressant)	Jolicoeur et al., 1977 [110]
Ethanol (CNS depressant)	Lester et al., 1970 [100]
Ethanol (CNS depressant)+cocaine (CNS stimulant)	Busse et al., 2005 [116]
Flurazepam (CNS depressant)	Vogel and Nathan, 1975 [108]
Heroin (analgesic)	Grigson et al., 2000 [117]
Heroin (analgesic)+cocaine (CNS stimulant)	Riley et al., 2019 [118]
Hexobarbital (CNS depressant)	Vogel and Nathan, 1975 [108]
Ketamine (hallucinogen)	Etscorn and Parson, 1979 [119]
l-Amphetamine (CNS stimulant)	Carey and Goodall, 1974 [120]
Lysergic acid diethylamide (LSD) (hallucinogen)	Parker, 1996 [121]
Methamphetamine (CNS stimulant)	Martin and Ellinwood, 1973 [122]
Mescaline (hallucinogen)	Cappell and LeBlanc, 1971 [101]
Methaqualone (sedative hypnotic)	Vogel and Nathan, 1975 [108]
Methyprylon (sedative hypnotic)	Jolicoeur et al., 1977 [110]
Methylone (synthetic cathinone; CNS stimulant)	Manke et al., 2021 [123]
Methylphenidate (CNS stimulant)	Riley and Zellner, 1978 [124]
Morphine (analgesic)	Cappell et al., 1973 [102]
Nicotine (CNS stimulant)	Etscorn, 1980 [125]
Pentobarbital (CNS depressant)	Buresova and Bures, 1980 [126]
Phencyclidine (PCP) (hallucinogen)	Etscorn and Parson, 1979 [119]
Phenobarbital (CNS depressant)	Vogel and Nathan, 1975 [108]
